# Understanding the Green Procurement Behavior of Household Appliance Manufacturing Industry: An Empirical Study of the Enablers

**DOI:** 10.1155/2023/9719019

**Published:** 2023-01-31

**Authors:** Fuli Zhou, Dongge Si, Sunil Tiwari

**Affiliations:** ^1^College of Economics and Management, Zhengzhou University of Light Industry, Zhengzhou, China; ^2^Department of Operations Management & Decision Science, ESSCA School of Management, Lyon, France

## Abstract

Green procurement, as a crucial green supply chain practice, contributes to sustainability achievement and reduces carbon emissions by selecting sustainable suppliers or outsourcing partners. The green procurement of household appliance manufacturing can reduce carbon emissions from the source and increase the competitiveness of products. To help better understand the driving powers and influential mechanism of green purchasing behavior for household appliance manufacturers, the green procurement mechanism is investigated by presenting an empirical study considering both endogenous and exogenous factors. A survey-based questionnaire is designed, and a semistructured interview is conducted for data collection. Besides, the structural equation model (SEM) approach is employed to test the supposed hypotheses and proposed assumptions based on the collected 529 questionnaire responses. The empirical results show that exogenous driving powers are more inclined to encourage household appliance manufacturers to perform green procurement strategy compared with endogenous factors. Additionally, the business strategy, governmental regulations, and customer awareness show greater influence on green purchasing behavior, while the corporate culture, production system, and suppliers have little impact. Taxation policies, environmental awareness, and green strategies are the three main driving factors for promoting green procurement from the governmental, individual, and organizational dimensions. This empirical study assists to investigate potential factors affecting green purchasing behavior and helps to disclose the influential mechanisms from a systematic viewpoint. Results derived from the empirical analysis could assist to achieve sustainability by better understanding green purchasing behavior and better promoting green procurement strategies.

## 1. Introduction

With the rapid development of the Chinese economy and the continuous advancement of urbanization, greenhouse gas emissions have increased significantly, and environmental pollution has become increasingly serious. The 20th National Congress of the Communist Party of China pointed out that we should accelerate the development mode's green transformation and promotes the formation of green and low-carbon modes of production and life. Environmental issues have received extensive attention from scholars worldwide [1–3], and consumers have gradually realized the importance of environmental protection. It is currently a hot topic to figure out how to cut carbon emissions, create a green economy, and achieve sustainable development of the environment, society, and economy [4, 5]. China's commitment to green and low-carbon development was reaffirmed when General Secretary Xi Jinping announced the target of reaching carbon neutrality by 2060 and reaching a carbon peak by 2030 at the United Nations General Assembly in September 2020. As carbon neutrality and carbon peaking have become important development strategies worldwide the future, manufacturing companies reliant on traditional supply chain management models are facing greater pressure for transformation. Conducting green supply chain management and improving environmental benefits have increasingly become development trends in many countries' manufacturing industries [6].

Different from the traditional supply chain management model, green supply chain management integrates the concepts of a full life cycle and producer responsibility in the supply chain to achieve green design, production, and circulation throughout the entire supply chain [7]. It is an innovative environmental management model in the context of new strategies [8]. It relies on the supply relationship between upstream and downstream enterprises, takes core enterprises as the fulcrum, and promotes upstream and downstream enterprises to improve their environmental performance and promote green innovation through green supplier management and green procurement, which in turn improves corporate performance [9]. A study found that there is a significant positive correlation between green procurement, green production, green recycling, corporate competitiveness, and environmental benefits [10]. The competition between enterprises has changed to the competition between supply chains, the relationship between upstream and downstream enterprises has become closer, and manufacturers are demanding more and more from their suppliers. Apple specified in its corporate social responsibility report that suppliers should provide green materials to reduce environmental impact. Dell, Ford, Toyota, and other multinational companies have also launched green procurement and production. To reduce environmental pollution, enterprises have started producing green products [11]. As the primary link in green product production, green procurement can improve the procurement efficiency of goods and services, reduce the negative impact on the environment, and achieve the same economic benefits in a more environmentally friendly way [12]. Therefore, more and more manufacturing enterprises have shifted their attention to green procurement, and some manufacturing enterprises have begun to actively implement the green procurement strategy, which has built a bridge between green production and green consumption.

At present, scholars have conducted extensive research on green procurement, including the factors that affect consumers' green procurement [13, 14], the application of green materials, and other aspects. The use of green materials in the construction industry or road construction can effectively improve the environmental performance of projects [15–20], which makes the selection of green suppliers key to green procurement [21–25]. In addition, the use of green logistics in the procurement process can effectively reduce operating costs, improve energy efficiency, and reduce carbon emissions [26–28]. Green manufacturing technology can integrate environmental impact and resource efficiency and is considered the future direction of modern manufacturing [29–32].

Additionally, scholars have also studied green procurement strategies in different industrial sectors, such as the oil, gas industry, real estate industry, and manufacturing industries [16, 33, 34]. The large amount of consumption potential and consumption capacity of household appliances make the green strategy more important due to its huge population base in the Chinese market. China is a large manufacturing country, the demand for household appliances is relatively large, and medium- and high-end household appliances are exported to several countries. Recently, the household appliance manufacturing industry has shown a development trend of green innovation, modernization, and intelligence [35], which has the following three development characteristics. First, household appliances are produced in large-scale, automated, and continuous production, with a large production scale and high per capita production capacity; second, household appliances are the comprehensive performance of new materials and technologies, and new materials and technologies in all walks of life are quickly applied to the household appliance industry; finally, products are diversified. With the increase in income level, people's requirements for high-quality living standards are becoming more and more intense. Household appliances are closely related to people's daily lives. Therefore, the characteristics of household appliances such as green environmental protection, pollution-free, safe, and intelligent have attracted much attention. People's demand for household appliances is the starting point of enterprise innovation. Household appliances are composed of many parts, and Chinese industrial plants pay more attention to assembly operations in the household appliance industry. Even though some brands can produce core parts, most of the components are outsourced, and they are usually assembled to be a product in an inefficient cost-effective way with high resource consumption. The green procurement is of great significance to carbon emission reduction and the sustainability achievement of the household appliance sector.

A better understanding of the influential ingredients of green procurement driving green purchasing behavior assists in green strategy promotion. Academic researchers and industrial practitioners have scrutinized the driving factors of green procurement. The results showed that external factors were more likely to prompt enterprises to conduct green procurement and that firms influenced by government regulations or regulatory measures will passively change their purchasing strategies [36]. Similarly, pressure from competitors would force companies to produce green products and thus change their purchasing strategies [37]. Most studies focused on external factors, such as governmental regulation, regional policy, and the requirements of its stakeholders. However, internal factors can also influence green purchasing. Corporate social responsibility, the attitude of executives [38], and concern for environmental friendliness [39] can also contribute to the implementation of green supply chain management.

China's household appliance manufacturers show an increasing trend in low-carbon, environmental protection, intelligent, and modern development. Many scholars have conducted academic research on green procurement in high-energy consumption industries; however, there is little research on disclosing the green procurement mechanism of the household appliance manufacturing industry. Besides, although there are extensive discussions on green procurement in previous publications regarding some industrial sectors, most researchers mainly focus on external drivers, including government policies and consumers, ignoring the internal factors of industrial organizations. However, under the prevailing philosophy of carbon reduction and sustainability achievement, household appliance manufacturer enterprises tend to show their internal impetus to perform green supply chain management practices. The green behaviors of manufacturing enterprises are not only motivated by external drivers (such as national regulations and social supervision) but are also driven by internal sustainability requirements. Therefore, this study tries to fill the gap by investigating the green procurement behavior of the household appliance manufacturing industry through quantitative research considering both external and internal drivers. The theoretical contributions of this research are as follows. First, a theoretical model is developed to address the green purchasing mechanism for the household appliance manufacturing industry considering comprehensive driving factors. The corporate culture is also involved in the novel framework, and related hypotheses are proposed based on the formulated theoretical model. Second, a quantitative study is performed and analyzed on the 529 questionnaire responses, which were collected by survey-based questionnaire and a semistructured interview. Third, the empirical study assists stakeholders in better understanding the green procurement behavior of household appliance manufacturers and contributes to green purchasing promotion and sustainability achievement by providing managerial insights for involved household appliance manufacturers, governments, suppliers, and consumers.

The rest of this paper is organized as follows: The literature review and research hypotheses are studied in Section 2. The research methodology and detailed steps are presented in Section 3. Research results are drawn and discussed in subsequent Section 4. Then, the theoretical and management implications are provided and discussed. Finally, we end the paper with conclusions.

## 2. Literature Review

### 2.1. Green Supply Chain Management

Green supply chain management (GSCM) is the integration of environmental thinking into all aspects of supply chain management [40, 41]. It has attracted more scholars' research as a business practice and emerging strategy [42–44], ecological innovation promotes the implementation of GSCM [45, 46]. GSCM can reduce waste and pollution in the entire supply chain and conduct product design, selection and procurement of raw materials, manufacturing, logistics and transportation, product sales, and other links with holistic thinking [47, 48]. Hsu et al. considered that GSCM includes three subsets of green procurement, environmental design, and green logistics [37]. Current research on supply chains focuses on the impact of GSCM on corporate performance. Some studies suggest that GSCM practices have positive effects on both environmental and financial performance [49–51]. On the contrary, Younis H et al. found that the subitems of GSCM had different impacts on corporate performance. They had no impact on environmental performance, but green procurement and environmental cooperation had significant effects on business performance [52]. Similarly, Geng et al. conducted a study on the relationship between GSCM and corporate performance in emerging Asian economies and found that GSCM has a positive effect on economic, environmental, operational, and social performance [53]. Additionally, customer pressure drives enterprises to conduct GSCM. Enterprises can control the environmental requirements of upstream procurement through environmental monitoring of suppliers, respond effectively to customer pressure, and form cooperative relationships with customers to improve financial performance [54]. Therefore, the implementation of green supply chain management plays a positive role in promoting enterprises. Green procurement as a key link in supply chain management can improve the operation and environmental performance of enterprises and make the products of those enterprises have stronger competitiveness.

### 2.2. Ingredients Affecting Green Procurement Behavior and Proposed Hypotheses

Green procurement, as the initial process of the sustainable supply chain, denotes that organizations prefer green suppliers with environmentally friendly products and services. It means that enterprises pay more attention to the green performances of their partners for environmental protection, resource conservation, and recycling in procurement activities. As an important part of GSCM, green procurement has attracted the research of many scholars. Research on green procurement of small- and medium-sized enterprises in developing countries found that green procurement has a positive impact on the competitiveness, business performance, environmental performance, and society of enterprises [34]. A comprehensive literature review of green procurement summarizes the internal and external drivers and obstacles of GSCM; the main driving factors are organizational factors, regulations, customers, competitors, and society, excluding suppliers [55]. Wang et al. believed that cost and customer factors affect the internal and external green practices of enterprises and improve environmental performance [56]. In contrast, Khodaparasti et al. argued that customer pressure is not significantly related to green purchasing and that environmental concerns, employee competencies, motivations, and rewards positively influence firms' green purchasing practices [57]. Besides, an empirical study by Ososanmi et al. showed that close collaboration between governments and other organizations and individuals can promote green supply chain practices in developing countries and that training can enhance awareness of sustainable development [58].

Scholars have different views on the driving factors of green purchasing. This paper puts forward to determine the factors that influence the green purchasing of enterprises from both internal and external aspects. The internal drives include business strategy, corporate culture, and production system, the external drives include government, suppliers, and consumers, and exogenous driving powers may affect endogenous driving powers, the dynamic model is shown in Figure 1.

First, business strategy is an active choice made by an enterprise to realize its long-term development goals and commercial value. Formulating a comprehensive and systematic business strategy is helpful to enhance the core competitiveness of an enterprise and stand out in the differentiated competition. The strategic level of the purchasing department and the environmental commitment level of the company drive the environmental performance of the enterprise, which in turn has a positive impact on purchasing performance [59]. Business strategy and corporate innovation have an inverted U-shaped relationship, and developing appropriate corporate strategies can have a positive impact on innovation performance [60]. Managers should create an environment conducive to sustainable development and commercial interests and classify the competitive environment through four strategies, including the company's industry structure, industry status, service market type, and capabilities. Using these four strategies, managers can optimize the economic returns on environmental investments and turn those investments into a competitive advantage [61]. In the research on the relationship between organizational innovation ability and green procurement implementation, it is found that organizational innovation ability will promotes the implementation of green procurement, and employees' commitment to change affects the implementation of green procurement [62]. From the company level, consumer purchasing behavior is positively related to the implementation of green procurement, and executive commitment is a key factor in green procurement and the development of green suppliers [63]. In addition to the positive impact of executives' commitment to green procurement, environmental cooperation with suppliers can indirectly affect green procurement [64].

Based on the above arguments, the following hypothesis is proposed as follows:

  H1: Business strategy significantly impacts the green procurement in the household appliance manufacturing industry.

Corporate culture is the soul of corporate development. An excellent corporate culture can create a good corporate environment, improve corporate cohesion and competitiveness, and thus promote corporate development. Corporate culture may reflect the uniqueness of an enterprise. It is an intangible factor to promote the innovation performance of enterprises [65]. Guiso et al. discussed the relationship between the dimensions of corporate culture and corporate performance and found that positive factors for corporate culture can improve corporate performance [66]. Therefore, although the corporate culture is invisible, it can exert a subtle influence on the enterprise.

Based on the above arguments, the following hypothesis is proposed as follows:

  H2: Corporate culture significantly impacts the green procurement of the household appliance manufacturing industry.

The production system is the core of the manufacturing enterprise and directly affects the quantity and quality of the enterprise's products. Progress and innovation in production technology are the driving forces for the economic development of the enterprise. An empirical study found that, compared with delivery time, cost, flexibility, and inventory optimization, factors such as product quality, production capacity, customer satisfaction, and supplier innovation have a greater positive influence on the benefits of sustainable supply management [67]. Products with high performance and a good experience are more likely to be favored by consumers [68]. Product packaging innovation is a part of ecological innovation, enterprises have gradually started to pay attention to packaging innovation, and the progress of production technology is conducive to the innovation of packaging ecological design and reducing the negative impact on brands [69]. Additionally, the lean practice of human technology can increase the innovation investment of enterprises, thereby improving the business performance of enterprises [70].

Based on the above arguments, the following hypothesis is proposed as follows:

  H3: Production systems significantly impact the procurement of the household appliance manufacturing industry.

The government can guide and restrain the behavior of enterprises, and government regulations and tax policies can promote the sustainable development of enterprises in purchasing and supply management [71–73]. The analysis of the green innovation practices factors of manufacturing supply chain management believes that there is a significant link between government regulation, stakeholder pressure, firm size, and green innovation practices [74]. Furthermore, production and start-up costs are the key factors that hinder the green production of enterprises and the most direct and effective way to stimulate the production of green products is to subsidize the production enterprises and gradually withdraw from the subsidy policies [5].

Based on the above arguments, the following hypothesis is proposed as follows:

  H4: Government significantly impacts the green procurement of the household appliance manufacturing industry.

Supplier selection is central to supply chain management. Research on the factors influencing supplier performance found that green supplier development is the moderating variable between green procurement and supplier performance [63]. When the supplier selection is determined through a multistage measurement standard, it is found that senior managers are willing to choose green suppliers, which will make the products of enterprises more environmentally friendly, thus improving the competitiveness of products and increasing the brand image of the company [75]. Establishing trust with suppliers is conducive to the development of a cooperative relationship. A good cooperative relationship can reduce the risk of the supply network, make the procurement system flexible, and ultimately improve customer satisfaction [76]. Additionally, an analysis of the determinants influencing the adoption of green procurement practices by Indian companies finds that internal environmental concerns, supplier collaboration, customer pressure, competitive pressure, and management support have a positive impact on green procurement [39].

Based on the above arguments, the following hypothesis is proposed as follows:

  H5: Suppliers have a significant impact on green procurement in the household appliance manufacturing industry.

The enhancement of environmental awareness makes consumers pay attention to the impact of products on the environment [77, 78]. Consumers are willing to pay more to buy green products, which are becoming a better choice. Based on a questionnaire survey and expert interviews, the key factors for strengthening the green procurement in the construction process are investigated, and it is found that, in addition to government regulations, bidding customer requirements are also key factors in green procurement [15]. Shen et al. believed that real estate developers in the Chongqing area of China lack an understanding of green procurement and green building materials and are unenthusiastic about producing green buildings. The main reasons for this phenomenon are the lack of consumer demand for green products and the lack of government incentives [16]. Similarly, an interview with senior managers found that managers generally believe that the implementation of sustainable supply chain management is related to growing customer expectations, and customer demand can effectively promote the company's sustainable supply chain management [79]. And when investigating the impact of environmental factors on consumer purchase intention, it was found that the purchase intention is highest when consumers can obtain both sustainable labeling and traceability information on products [80].

Based on the above arguments, the following hypothesis is proposed as follows:

  H6: Consumers significantly impact the green purchasing power of household appliance manufacturing.

Furthermore, the following relationships are assumed to exist between the various factors:

  H7: Business strategy has a significant impact on corporate culture.
  H8: Business strategy has a significant impact on the production system.
  H9: Corporate culture has a significant impact on the production system.
  H10: Suppliers have a significant influence on the production system.
  H11: Government has a significant influence on corporate culture.
  H12: Government has a significant influence on consumers.

Finally, a conceptual model and hypotheses on purchasing behavior are established Figure 2.

## 3. Methodology

### 3.1. Sample Design and Data Collection

Based on the above research assumptions and theoretical models, a questionnaire was designed to collect data. All measurements are taken from relevant research, and the wording was slightly modified to ensure that all items can be understood in this research. The questionnaire was divided into two parts. One is to count the information on the interviewees; the other is to investigate the driving factors affecting green procurement in the household appliance manufacturing industry. The 5-level Likert scale was used to design the questions. The survey objects were purchasing staff, sales staff, and academic staff, and the main method was an online questionnaire. Among the respondents, 53% were males and 47% were females, and the ratio of the two was similar. In terms of academic qualifications, most of the respondents have an associate degree or above in education. The respondents with a monthly income of 4000–5999 yuan accounted for the highest proportion (48.6%). Nearly half of the respondents were between the ages of 31 and 40 (46.2%).

The sample size required for this study was calculated from the desired level of 5–10 observations per parameter in structural equation modeling (SEM) [81]. A total of 26 measurement indicators were selected for this paper. To obtain more stable results, the questionnaires were sent to 529 subjects, and all of them were received. Finally, before data analysis, the questionnaire was screened, and invalid questionnaires were eliminated. The total number of valid questionnaires was 517, with an effective rate of 97.7%, indicating that the overall effect of completing the questionnaire was good.

### 3.2. Variables and Measurement Scales

The green purchasing power of enterprises consists of endogenous power and exogenous power, in which endogenous power refers to the process of the effect of the characteristics of the household appliance manufacturing industry on green purchasing behavior, it includes three categories: business strategy, corporate culture, and production system. Exogenous motivation mainly includes three factors: government, suppliers, and consumers. The definitions and measurements for this study are described in the following.

#### 3.2.1. Business Strategy

Under the guidance of the sustainable development concept, enterprises must develop a green development strategy and take it as a long-term guidance strategy if they want to achieve long-term development goals. The measurement of “Business strategy” includes five items in Table 1.

#### 3.2.2. Corporate Culture

Excellent corporate culture can guide and motivate employees to work better, improve the cohesion of the company, and promote the company to develop in a better direction. The measurement of “Corporate culture” includes three items in Table 1.

#### 3.2.3. Production System

The production system is divided into two aspects. One is the software aspect, namely the construction of technology, systems, organization, and management; the second is hardware, involving equipment investment, operation, maintenance, and so on. The production system of the household appliance manufacturing industry should be based on green production. The measurement of “Production system” includes three items in Table 1. In Table 1, there are three items to measure the green procurement driving force of the household appliance manufacturing industry.

#### 3.2.4. Government

The government can promote enterprises to conduct green procurements through economic, administrative, legal, and other means. Simultaneously, the government should take the initiative to implement green procurement, give play a role of demonstrative and guidance, and promote enterprises to produce green products. The measurement of “Government” includes four items in Table 1.

#### 3.2.5. Supplier

Supplier management is an important part of green procurement. A scientific supply structure and stable cooperative relationships are conducive to reducing risks and enhancing corporate competitiveness. The measurement of “Suppliers” includes four items in Table 1.

#### 3.2.6. Consumer

With the increasing awareness of environmental protection, consumers will make more green choices when choosing products and consumption methods [82]. Simultaneously, suppliers have received the “green demand” signal from the market, which prompted the production company to develop its business strategy in a green direction. The measurement of “Consumers” includes four items in Table 1.

In summary, there are 11 measurement indicators for endogenous latent variables that affect the green purchasing driving powers of the household appliance manufacturing industry, 12 measurement indicators for exogenous latent variables, and 3 measurement indicators for measuring green purchasing driving powers, as shown in Table 1.

### 3.3. Descriptive Statistical Analysis

After sorting out the questionnaire data, descriptive statistical analysis was conducted on the mean, standard deviation, skewness, kurtosis, and factor loading to ensure the applicability of the data. The statistical results are shown in Table 2.

From the average values of various measurement indicators in Table 2, it can be seen that the attitude of the respondents tends to be between “average” and “strongly agree” and the overall attitude is relatively positive. In addition, the skewness and kurtosis of the data were analyzed to test whether the data conformed to a normal distribution, and found that the sample data conformed to a normal distribution. In addition, the factor loading is basically above 0.6, indicating that the basic fitness of the model is good and can be used for subsequent analysis.

## 4. Empirical Results

### 4.1. The Results of the Measurement Model

To verify the measurement model, reliability and validity analyzes were carried out. Reliability was evaluated by Cronbach's alpha. In this study, the test results of the Cronbach's alpha coefficient for the 26 measurement indicators of green purchasing dynamics in the household appliance manufacturing industry are shown in Table 3.

Table 3 shows that the overall reliability value of the 26 measured variables on the scale reaches 0.922, which indicates that the questionnaire survey in this study has excellent reliability.

By analyzing the test values of KMO and Bartlett's, it is determined whether the sample data is suitable for factor analysis, and its validity is verified. The results are shown in Table 4.

Table 4 shows that the value of KMO is between 0.9 and 1.0, indicating that the correlation of the sample data is excellent. Among them, the significance is 0.000, less than 0.001, indicating that the sample data have good construct validity and can be used for factor analysis.

### 4.2. The Results of the Full Model

Amos is used to import the questionnaire data into the structural equation model of the dynamic mechanism, and the unstandardized regression coefficients estimated using the maximum likelihood method are shown in Table 5. In SEM analysis, judging whether the influence between variables is significant is based on the critical ratio C.R. If the absolute value of C.R. is greater than 1.96, the parameter estimate will reach the significance level of 0.05.

As shown in Table 5, the absolute value of the influence of corporate culture, production system, and suppliers on the green purchasing dynamic of the household appliance manufacturing industry is less than 1.96, and the *P* value is all greater than 0.05. Although other path coefficients are significant, the impact effect has not yet reached a significant level. The intrinsic quality of the model is acceptable.  Table 6 shows the fit of the initial model.

Table 6 shows that the output values of all fitting indices are in line with the standard except that the chi-square freedom degree ratio is too large and the GFI value is too low. In order to make the hypothetical model better fit the sample data, it is necessary to revise the model.

This paper will make corrections based on the value of the modification indices (MI). The specific correction method is to gradually select the two paths with the largest MI value, correlate them, and reduce the corresponding chi-square value, thus reducing the proportion of chi-square degrees of freedom. However, in the correction process, the maximum MI value cannot be blindly selected, because it is necessary to ensure that there is practical significance between the two connected measurement variables. Therefore, according to this method, the SEM is modified in this paper as follows.

From the results of the model, the MI value between e16 and e26 is the largest. If the residual correlation path between them increases, the chi-square value will decrease significantly, and the degree of freedom of the model will also decrease. In addition, from a practical perspective, there are also correlation between suppliers' production of green materials and the household appliance manufacturing industry's initiative to promote a green purchasing strategy. Therefore, we can consider adding correlation paths between e16 and e26, connecting them with two-way arrows, and rerunning the model. If the fitting effect is not good, repeat the above method until the model fits well. After repeated corrections, the following model is obtained, as shown in Figure 3.

The revised model fitting index and model path coefficient are shown in Tables 7 and 8, respectively.

It can be seen from Table 7 that all fitting indexes meet the requirements, indicating that the model fits well.

From Table 8, the effect of business strategy on green procurement is 0.095, the C.R. and *P* values meet the conditions, so the impact is significant, and H1 is supported. Similarly, the government's influence on green purchasing is 0.934, the C.R. and *P* values satisfy the conditions, and the influence is significant. H4 is supported; the influence of consumers on green procurement is 0.298, C.R., and *P* values satisfy the conditions, so the influence is significant, and H6 is supported. In addition, the C.R. and *P* values of corporate culture, the production system, and suppliers did not meet the requirements, so H2, H3, and H5 were not verified. In addition, H7, H8, H9, H10, and H12 have also been verified, indicating that there is indeed a significant impact between the driving factors.

Based on the previous analysis, the path coefficient is used to calculate the impact of each measurement variable on the green purchasing dynamic of the household appliance manufacturing industry, and the results of the green purchasing dynamic mechanism of the household appliance manufacturing industry are explained. The calculation results of the path coefficient are shown in Table 9.

According to Table 9, among the five measurement variables that constitute a corporate strategy, green development strategy and green marketing strategy have a greater impact on household appliance manufacturing, followed by the other three factors; among the government factors, tax policy has the greatest impact on enterprises' green purchasing behavior, while the other three factors have positive effects, but the degree of influence is not much different. Among the measured variables of consumers, the improvement in consumers' awareness of environmental protection and living standards significantly impacted the green purchasing power of the household appliance manufacturing industry, which is higher than the other two measured variables.

## 5. Discussion and Implications

At present, many scholars have conducted research on the green procurement activities that drive the real estate industry and the cosmetics industry, but there are few studies on the driving factors that drive green procurement in the household appliance manufacturing industry. As a large manufacturing country, China's household appliance manufacturing industry is mature and competitive. In recent years, the proportion of medium- and high-end products exported has increased significantly. The household appliance manufacturing industry can develop and create new products while meeting the basic needs of many countries. Under the international environmental protection requirements and China's carbon emission reduction target, it is very important to promote green and low-carbon products and accelerate the green transformation of the household appliance manufacturing industry. The green purchasing behavior of the household appliance manufacturing industry can reduce carbon emissions at the source and help enterprises to produce green products. In addition, procurement activities are the beginning of the supply chain and the source of corporate environmental management. Its significance has long been recognized by many internationally renowned companies. If the Chinese household appliance manufacturing industry wants to gain a foothold in the fierce market competition, it is crucial to implement a green procurement strategy.

Based on the extensive literature reading, this study combined with household appliance manufacturing is in urgent need of the actual situation of the green transformation, constructing an evaluation index system of green purchasing power appliances manufacturing. The research hypotheses are tested through questionnaire data, and the internal and external factors affecting the green procurement of household appliance enterprises are analyzed. Our study provides empirical evidence for driving green purchasing in the appliance manufacturing industry in the context of corporate green transformation. First, external factors have a more significant contributing relationship for firms compared to internal factors. Government regulations, consumer attitudes, and business strategies have significant effects on green procurement, while suppliers, corporate culture, and production systems have insignificant effects on green procurement. These findings complement earlier work on internal and external factors [39, 57], which emphasizes the importance of government regulations, consumer attitudes, and business strategies.

Second, this paper fills the previous literature gap by analyzing the upstream and downstream of the supply chain and assuming that suppliers and customers are the driving factors for implementing green procurement [83]. Additionally, this study analyzes the effects of each influencing factor and its subdivision elements to help each internal and external stakeholder find specific ways to promote green procurement in enterprises.

Finally, the reward and punishment policies imposed by the government can change the production strategies of firms, especially in light of green and low-carbon environmental requirements, which compel firms to make a green transition. Similarly, consumer demand is the driving force of enterprise production. Low-carbon and environmentally friendly products are more likely to be favored by consumers, thus increasing firms' motivation to implement green implementation. But this result was contrary to Khodaparasti et al., who concluded that pressure from customers is not significantly related to firms' green purchasing behavior [57]. The various green strategies implemented by companies can improve their market competitiveness and increase their confidence in green procurement.

Additionally, we also offer some explanations for the insignificance of the hypothesized effects. Compared to corporate strategy, the influence of corporate culture may be smaller, and technological innovation strategies may be better than updating and improving production technology and production processes. The findings also found that suppliers do not promote green purchasing in firms, which contrasts with previous studies; specifically, Ghosh found a positive effect of supplier collaboration on green purchasing [39].

### 5.1. Theoretical Implications

This paper contributes to green supply chain management by providing insights into a better understanding of green procurement behavior in the Chinese household appliance manufacturing industry. Previous studies have conducted in-depth analysis and research on the driving factors of green procurement in different industries, but few scholars have researched the driving factors of green procurement in the household appliance manufacturing industry. Therefore, this article aims to extract the driving factors that affect the green purchasing dynamics of the household appliance manufacturing industry by referring to a large number of documents. On this basis, research hypotheses are proposed, theoretical models are constructed, data are obtained using questionnaire surveys, and key factors driving the implementation of green procurement in the household appliance manufacturing industry are identified with the help of Amos software, which can provide references for related theoretical research.

### 5.2. Managerial Implications

A better understanding of the driving factors affecting green procurement enlightens industrial managers to perform green procurement strategies for the household appliance manufacturing industry. Besides, the stakeholders will also benefit from this study. For household appliance manufacturing enterprises, it will help enterprises formulate targeted strategies to improve the construction of enterprise-related systems, help enterprises produce green products, technological innovation, reduce environmental pollution, and further improve their economic and environmental benefits, and enhance enterprise product market competitiveness and corporate influence. Our study will help the government to expand the scope of the green material list, provide preferential policies and product standards, and improve relevant laws and regulations that will help enterprises implement green procurement. For suppliers, a better understanding of the influential mechanisms of green procurement would motivate the green supplier to develop green manufacturing technologies and improve the authoritative material certification system. The countermeasures also can be made to promote green procurement and green consumption based on the discovered influential mechanism.

## 6. Conclusions

In the context of green and high-quality development, this study establishes a model of the relationship between internal and external factors and green procurement in the household appliance manufacturing industry to investigate the motivations behind enterprises' green procurement behavior and hasten the green transformation of enterprises in the procurement process. Through the above empirical analysis, this study shows that, among the six factors that affect the green purchasing dynamic of the household appliance manufacturing industry, government, consumer, and business strategy have a significant impact on it; however, the influence of corporate culture, production system, and supplier factors is not significant. But its practical significance cannot be denied. Government factors have the most significant impact on the green purchasing dynamics of the household appliance manufacturing industry, which indicates that government support will greatly promote green procurement by household appliance manufacturers. The influence of consumer factors on the green purchasing dynamics of the household appliance manufacturing industry guides companies to produce green products to a certain extent. Corporate strategy is less important than the other two, but it is also very important. Therefore, enterprises should not only improve their green procurement capabilities but also pay close attention to the government's various low-carbon policies and improve their ability to adapt to changes in procurement and manufacturing. In addition, enterprises should also pay attention to the environmental needs of consumers and produce more low-carbon and environmentally friendly products.

From their respective measurement variables, among the government factors that have the most significant impact on the green purchasing dynamics of the household appliance manufacturing industry, there are preferential policies such as fiscal and taxation. This indicates that household appliance manufacturers need strong support from preferential policies to implement green procurement strategies. Among the consumer factors, the improvement of living standards has the greatest influence on the green purchasing dynamics of the household appliance manufacturing industry. This indicates that with the improvement of people's living standards, people are more inclined to choose energy-saving, environmentally-friendly, green, and safe products, especially household items closely related to daily life. Among the corporate strategic factors, the influence of green development strategy and green marketing strategy on the green procurement dynamics of the household appliance manufacturing industry is consistent, indicating that green development is a development concept that enterprises must follow in the future.

However, this research also has some limitations. First, the influential factors were based on internal and external categories, based on previous studies to expand the selection. However, green procurement may also be driven by other company-specific factors. Future research could tap into some other potential factors, such as the influence of competitors. Additionally, the sample size using the questionnaire method is limited. Diversified sample or data mining techniques can also be employed to enrich the sample data in future research, which will increase the statistical dynamics of the results and draw more specific conclusions.

## Figures and Tables

**Figure 1:** Theoretical model of green purchasing mechanism.

**Figure 2:** Conceptual model of green procurement drives mechanism in household appliance manufacturing.

**Figure 3:** Correction path diagram of structural equation model of green purchasing power mechanism of household appliance manufacturing industry.

**Table 1:** Green procurement driving powers index system.

Classifications	Latent variables	Codes	Measure variables
Endogenous latent variables	Business strategy (*η*_1_)	*y*_1_	Senior leadership support
		*y*_2_	Green marketing strategy
		*y*_3_	Technological innovation
		*y*_4_	Green development strategy
		*y*_5_	Improve the competitiveness of enterprises
	Corporate culture (*η*_2_)	*y*_6_	Green corporate culture
		*y*_7_	Green education for purchasing staff
		*y*_8_	Green management systems
	Production system (*η*_3_)	*y*_9_	Environmentally friendly production process
		*y*_10_	Waste recycling system
		*y*_11_	Energy-saving and consumption-reducing production technology
	Green procurement driving powers (*η*_4_)	*y*_12_	Actively implement green procurement strategy
		*y*_13_	Actively organize green procurement activities
		*y*_14_	Actively publicity green procurement strategy

Exogenous latent variables	Government (*ξ*_1_)	*x*_1_	Fiscal, tax, and other preferential policies
		*x*_2_	Strict penalty policy
		*x*_3_	Develop green product standards
		*x*_4_	The guidance of government green procurement
	Suppliers (*ξ*_2_)	*x*_5_	Suppliers produce green materials
		*x*_6_	Scientific supply structure
		*x*_7_	Stable supply chain alliance relationship
		*x*_8_	Authoritative green material certification system
	Consumers (*ξ*_3_)	*x*_9_	Consumer environmental awareness
		*x*_10_	Improvement of living standards
		*x*_11_	Demand for green products
		*x*_12_	Green consumption preference

**Table 2:** Data descriptive statistics.

Variable names	Measurement item	Mean	Standard deviation	Skewness	Kurtosis	Factor loading
Business strategy (*η*_1_)	*y*_1_	4.10	1.029	−0.885	−0.253	0.605
	*y*_2_	4.04	0.796	−0.655	0.171	0.764
	*y*_3_	4.06	0.842	−0.598	−0.281	0.678
	*y*_4_	4.07	0.847	−0.703	−0.039	0.773
	*y*_5_	3.99	0.834	−0.646	0.010	0.711

Corporate culture (*η*_2_)	*y*_6_	4.05	1.032	−1.092	0.693	0.565
	*y*_7_	4.17	0.833	−0.828	0.143	0.652
	*y*_8_	4.22	0.790	−0.902	0.534	0.619

Production system (*η*_3_)	*y*_9_	4.17	0.819	−0.671	−0.308	0.553
	*y*_10_	4.09	0.785	−0.585	−0.061	0.666
	*y*_11_	4.19	0.827	−0.960	0.662	0.725

Green procurement driving powers (*η*_4_)	*y*_12_	4.03	1.109	−1.077	0.420	0.712
	*y*_13_	4.21	0.957	−1.289	1.413	0.671
	*y*_14_	4.17	0.890	−0.999	0.728	0.662

Government (*ξ*_1_)	*x*_1_	4.29	0.831	−0.992	0.253	0.644
	*x*_2_	4.01	0.864	−0.533	−0.445	0.625
	*x*_3_	4.10	0.794	−0.628	−0.039	0.644
	*x*_4_	4.05	0.824	−0.573	−0.234	0.674

Suppliers (*ξ*_2_)	*x*_5_	4.20	0.851	−0.726	−.387	0.605
	*x*_6_	4.04	0.772	−0.575	0.114	0.818
	*x*_7_	4.08	0.784	−0.646	0.154	0.727
	*x*_8_	4.26	0.829	−0.958	0.254	0.616

Consumer (*ξ*_3_)	*x*_9_	4.13	0.988	−0.960	0.053	0.664
	*x*_10_	4.16	0.806	−0.720	0.108	0.646
	*x*_11_	4.21	0.809	−0.777	−0.037	0.712
	*x*_12_	4.17	0.762	−0.606	−0.114	0.670

**Table 3:** Reliability analysis of sample data.

Cronbach's alpha	Cronbach's alpha based on standardized terms	Number of terms
0.922	0.926	26

**Table 4:** KMO and Bartlett's test.

KMO		0.925
Bartlett's test	Approximate chi-square	3879.780
	Degree of freedom	325
	Statistical significance	0.000

**Table 5:** Initial model path coefficient table.

Path			Estimate	S.E.	C.R.	*P*
GP driving powers	←	Business strategy	0.129	0.039	3.309	^*∗∗∗*^
GP driving powers	←	Corporate culture	−0.115	0.094	−1.230	0.219
GP driving powers	←	Production system	−0.098	0.118	−.829	0.407
GP driving powers	←	Government	0.975	0.217	4.499	^*∗∗∗*^
GP driving powers	←	Consumer	0.000	0.062	−0.004	0.997
GP driving powers	←	Supplier	0.332	0.115	2.895	0.004
Corporate culture	←	Business strategy	0.200	0.024	8.244	^*∗∗∗*^
Production system	←	Business strategy	0.150	0.020	7.508	^*∗∗∗*^
Production system	←	Corporate culture	0.162	0.021	7.829	^*∗∗∗*^
Production system	←	Supplier	0.135	0.018	7.462	^*∗∗∗*^
Corporate culture	←	Government	0.181	0.210	8.542	^*∗∗∗*^
Consumer	←	Government	0.025	0.009	2.743	0.006
Improve the competitiveness of enterprises	←	Business strategy	1.000			
Green development strategy	←	Business strategy	1.075	0.068	15.824	^*∗∗∗*^
Technological innovation	←	Business strategy	0.948	0.067	14.162	^*∗∗∗*^
Green marketing strategy	←	Business strategy	1.000	0.064	15.670	^*∗∗∗*^
Senior leadership support	←	Business strategy	1.010	0.081	12.412	^*∗∗∗*^
Green management system	←	Corporate culture	1.000			
Green education for purchasing staff	←	Corporate culture	1.066	0.105	10.192	^*∗∗∗*^
Green corporate culture	←	Corporate culture	1.054	0.120	8.806	^*∗∗∗*^
Energy-saving and consumption-reducing production technology	←	Production system	1.000			
Waste recycling system	←	Production system	0.968	0.098	9.922	^*∗∗∗*^
Environmentally friendly production process	←	Production system	0.998	0.101	9.830	^*∗∗∗*^
The guidance of government GP	←	Government	1.000			
Develop green product standards	←	Government	0.924	0.094	9.867	^*∗∗∗*^
Strict penalty policy	←	Government	0.933	0.100	9.333	^*∗∗∗*^
Fiscal, tax, and other preferential policies	←	Government	1.567	0.117	13.338	^*∗∗∗*^
Authoritative green material certification system	←	Supplier	1.000			
Stable supply chain alliance relationship	←	Supplier	1.085	0.086	12.577	^*∗∗∗*^
Scientific supply structure	←	Supplier	1.203	0.091	13.250	^*∗∗∗*^
Suppliers produce green materials	←	Supplier	0.983	0.089	11.054	^*∗∗∗*^
Actively implement GP strategy	←	GP driving powers	1.000			
Actively organize green procurement activities	←	GP driving powers	3.037	0.553	5.492	^*∗∗∗*^
Actively publicity GP strategy	←	GP driving powers	1.359	0.278	4.886	^*∗∗∗*^
Green consumption preference	←	Consumer	1.000			
Demand for green products	←	Consumer	1.085	0.090	12.086	^*∗∗∗*^
Improvement of living standards	←	Consumer	1.109	0.090	12.319	^*∗∗∗*^
Consumer environmental awareness	←	Consumer	1.193	0.096	12.490	^*∗∗∗*^

*Note*. GP = green procurement. SE = standard error. C.R. = critical ratio. *P* < 0.001^*∗∗∗*^.

**Table 6:** Initial model fitting index.

Index	*χ*2/d*f*	RMSEA	CFI	ILI	NFI	GFI
Reference	<5	<0.08	>0.9	>0.9	>0.9	>0.9
Output value	5.73	0.072	0.921	0.918	0.957	0.836

**Table 7:** Modified model fit index.

Index	*χ*2/d*f*	RMSEA	CFI	ILI	NFI	GFI
Reference	<5	<0.08	>0.9	>0.9	>0.9	>0.9
Output value	3.71	0.053	0.921	0.935	0.959	0.917

**Table 8:** Corrected model path coefficient.

Path			Estimate	S.E.	C.R.	*P*
GP driving powers	←	Business strategy	0.095	0.030	3.158	0.002
GP driving powers	←	Corporate culture	-0.047	0.070	-0.677	0.498
GP driving powers	←	Production system	-0.100	0.071	-1.407	0.159
GP driving powers	←	Government	0.934	0.196	4.766	^*∗∗∗*^
GP driving powers	←	Consumer	0.298	0.095	3.145	0.002
GP driving powers	←	Supplier	0.003	0.035	0.089	0.929
Corporate culture	←	Business strategy	0.204	0.024	8.459	^*∗∗∗*^
Production system	←	Business strategy	0.226	0.026	8.798	^*∗∗∗*^
Production system	←	Corporate culture	0.234	0.026	8.968	^*∗∗∗*^
Production system	←	Supplier	0.234	0.026	9.004	^*∗∗∗*^
Corporate culture	←	Government	0.005	0.008	0.597	0.550
Consumer	←	Government	0.176	0.021	8.419	^*∗∗∗*^
Improve the competitiveness of enterprises	←	Business strategy	1.000			
Green development strategy	←	Business strategy	1.074	0.068	15.805	^*∗∗∗*^
Technological innovation	←	Business strategy	0.915	0.065	14.033	^*∗∗∗*^
Green marketing strategy	←	Business strategy	1.008	0.064	15.783	^*∗∗∗*^
Senior leadership support	←	Business strategy	1.012	0.081	12.421	^*∗∗∗*^
Green management system	←	Corporate culture	1.000			
Green education for purchasing staff	←	Corporate culture	1.052	0.092	11.391	^*∗∗∗*^
Green corporate culture	←	Corporate culture	1.026	0.108	9.470	^*∗∗∗*^
Energy-saving and consumption-reducing production technology	←	Production system	1.000			
Waste recycling system	←	Production system	0.973	0.079	12.389	^*∗∗∗*^
Environmentally friendly production process	←	Production system	0.920	0.078	11.749	^*∗∗∗*^
The guidance of government GP	←	Government	1.000			
Develop green product standards	←	Government	0.907	0.094	9.688	^*∗∗∗*^
Strict penalty policy	←	Government	0.958	0.102	9.370	^*∗∗∗*^
Fiscal, tax, and other preferential policies	←	Government	1.625	0.123	13.249	^*∗∗∗*^
Authoritative green material certification system	←	Supplier	1.000			
Stable supply chain alliance relationship	←	Supplier	1.045	0.077	13.635	^*∗∗∗*^
Scientific supply structure	←	Supplier	1.074	0.076	14.078	^*∗∗∗*^
Suppliers produce green materials	←	Supplier	0.771	0.069	11.108	^*∗∗∗*^
Actively implement GP strategy	←	GP driving powers	1.000			
Actively organize green procurement activities	←	GP driving powers	3.070	0.553	5.552	^*∗∗∗*^
Actively publicity GP strategy	←	GP driving powers	1.271	0.257	4.955	^*∗∗∗*^
Green consumption preference	←	Consumer	1.000			
Demand for green products	←	Consumer	1.029	0.086	11.946	^*∗∗∗*^
Improvement of living standards	←	Consumer	1.159	0.094	12.385	^*∗∗∗*^
Consumer environmental awareness	←	Consumer	1.205	0.098	12.258	^*∗∗∗*^

*Note.* GP = green procurement. SE = standard error. C.R. = critical ratio. *P* < 0.001^*∗∗∗*^.

**Table 9:** The effects of relationship between each group of measurement variables and green purchasing drives.

Latent variables	Coefficient	Measure variables	Coefficient	result
Business strategy	0.225	Senior leadership support	0.594	0.134
		Green marketing strategy	0.765	0.172
		Technological innovation	0.666	0.150
		Green development strategy	0.766	0.172
		Improve the competitiveness of enterprises	0.724	0.163

Corporate culture	−0.096	Green corporate culture	0.513	−0.049
		Green education for purchasing staff	0.652	−0.063
		Green management system	0.658	−0.063

Production system	−0.215	Environmentally friendly production process	0.617	−0.133
		Waste recycling system	0.674	−0.145
		Energy-saving and consumption-reducing production technology	0.657	−0.141

Government	1.631	Fiscal, tax, and other preferential policies	0.868	1.416
		Strict penalty policy	0.492	0.802
		Develop green product standards	0.508	0.829
		The guidance of government green procurement	0.538	0.877

Supplier	0.007	Suppliers produce green materials	0.526	0.004
		Scientific supply structure	0.773	0.005
		Stable supply chain alliance relationship	0.732	0.005
		Authoritative green material certification system	0.664	0.005

Consumer	0.571	Consumer environmental awareness	0.689	0.393
		Improvement of living standards	0.700	0.400
		Demand for green products	0.636	0.363
		Green consumption preference	0.638	0.364

## Data Availability

The data used to support the findings of this study are available from the corresponding author upon request.
